The article "Targeting BET bromodomain proteins in solid tumors" was published in 2016. Journal: Oncotarget.

# Targeting BET bromodomain proteins in solid tumors

**DOI:** 10.18632/oncotarget.9804

**Published:** 2016-06-05

**Authors:** Vaibhav Sahai, Amanda J. Redig, Katharine A. Collier, Frank D. Eckerdt, Hidayatullah G. Munshi

**Affiliations:** ^1^ Department of Medicine, University of Michigan Medical Center, Ann Arbor, MI, USA; ^2^ Dana-Farber Cancer Institute and Harvard Medical School, Boston, MA, USA; ^3^ Department of Medicine, Feinberg School of Medicine, Northwestern University, Chicago, IL, USA; ^4^ The Robert H. Lurie Comprehensive Cancer Center of Northwestern University, Chicago, IL, USA; ^5^ Jesse Brown VA Medical Center, Chicago, IL, USA

**Keywords:** NUT midline carcinoma, breast and prostate cancers, lung cancers, gastrointestinal cancers, brain tumors

## Abstract

There is increasing interest in inhibitors targeting BET (bromodomain and extra-terminal) proteins because of the association between this family of proteins and cancer progression. BET inhibitors were initially shown to have efficacy in hematologic malignancies; however, a number of studies have now shown that BET inhibitors can also block progression of non-hematologic malignancies. In this Review, we summarize the efficacy of BET inhibitors in select solid tumors; evaluate the role of BET proteins in mediating resistance to current targeted therapies; and consider potential toxicities of BET inhibitors. We also evaluate recently characterized mechanisms of resistance to BET inhibitors; summarize ongoing clinical trials with these inhibitors; and discuss potential future roles of BET inhibitors in patients with solid tumors.

## INTRODUCTION

Epigenetic changes that occur during cancer progression are increasingly recognized as a potential target for therapeutic intervention. Bromodomains (BRDs) are evolutionarily conserved protein interaction modules that bind to acetylation motifs present in histones and enable recruitment of transcription factors and other chromatin regulators during the precise sequence of events involved with RNA transcription [1, 2]. The BET (BRD and extra-terminal) family of proteins regulates the transcription of genes involved in several human diseases and includes family members BRD2, BRD3, BRD4, and the testis-specific BRDT [1, 2]. Significantly, BRD4 has been established as a key regulator of transcriptional elongation by recruiting the positive transcription elongation factor b (P-TEFb) complex to chromatin [3, 4]. BRD4 also mediates the formation of the active form of P-TEFb, which in turn phosphorylates and activates RNA polymerase II (RNA Pol II; Figure 1). BRD4 is enriched in large numbers of enhancer regions, and also in some large super-enhancer regions, and mediates expression of key transcription factors important for cancer development and progression [5]. BET inhibition displaces BRD4 from these super-enhancers and blocks expression of certain key oncogenes, such as MYC [5]. Besides binding histones, BRD proteins can also regulate cellular function by binding to a number of other proteins (Table 1) [1, 2, 6-11].

**Figure 1:** Transcriptional activation by BRD4 Binding of BRD4 to acetylated histones recruits the positive transcription elongation factor b (P-TEFb) complex to chromatin. BRD4 also mediates activation of P-TEFb, which in turn phosphorylates and activates RNA polymerase II (RNA Pol II) to initiate gene transcription.

Significantly, a number of selective and potent small-molecule inhibitors have been developed that can compete with the acetyl-binding pockets present in the bromodomains of BET proteins and block gene expression (Figure 2) [1, 2]. These compounds were initially shown to be effective in the treatment of leukemia, lymphoma, and multiple myeloma, primarily as a result of repressing c-MYC expression [1, 12, 13]. Further investigation has now shown that BET inhibitors can repress expression of oncogenic transcription factors beyond c-MYC, thus expanding their potential clinical utility to include solid tumors [14-16]. Interested readers are referred to recent Reviews for additional details on the mechanisms by which BET proteins regulate gene transcription [3, 4, 17]*.* In this Review, we outline the efficacy of BET inhibitors in select solid tumors; summarize the role of BET proteins in mediating resistance to current targeted therapies; and consider potential toxicities of BET inhibitors. We also evaluate recently characterized mechanisms of resistance to BET inhibitors; summarize ongoing clinical trials with these inhibitors; and discuss potential future roles of BET inhibitors in patients with solid tumors.

**Table 1:** Interactions of BET proteins with other proteins

Protein	Effect of interaction	References
Acetylated Histones	Regulate gene expression (e.g., MYC)	[1, 2]
P-TEFb	Dissociate HEXIM1 to activate P-TEFb	[6]
Cyclin-T1	Stabilize BRD4/P-TEFb complex to enable activation of P-TEFb-responsive genes	[6]
RelA	Prevent degradation of RelA to maintain active form of NF-κB	[7]
TWIST	Regulate WNT5A expression to promote invasion, cancer stem cell-like properties and tumorigenesis	[8]
GATA1	Promote chromatin occupancy at erythroid target genes to regulate erythroid maturation	[9]
Androgen Receptor (AR)	Transcriptional regulation of AR target genes	[10]
WHSC1	Regulate ERα expression and function	[11]

**Figure 2:** Binding of BET family proteins (BRD2, BRD3, BRD4 and BRDT) to acetylated (Ac) histones regulates expression of genes that contribute to cancer progression Small-molecule inhibitors, such as JQ1, compete with the acetyl-binding pockets present in the bromodomains of BET proteins and block BET-dependent gene expression.

## TREATMENT OF SELECT SOLID TUMORS WITH BET INHIBITORS

### BET inhibitors and NUT midline carcinoma

Human BRD4 was initially identified because of its role in NUT midline carcinoma (NMC) [18, 19], a rare subtype of squamous cell carcinoma characterized by a translocation most often involving the *NUT* gene and BRD4 [20]. Other potential translocation partners also include BRD3 [18, 19]. NMC typically arises from the midline structures of the head, neck, and thorax, and can be diagnosed in both pediatric and adult patients [20]. The disease is extremely aggressive with both locoregional and distant spread, and median overall survival (OS) was reported at 6.7 months in one large series [20]. Mechanistically, the BRD4-NUT fusion protein blocks differentiation of NMC cells partly through expression of c-MYC [21]. Treatment of NMC cells with BET inhibitors results in proliferation arrest and squamous cell differentiation *in vitro* and in mouse xenograft models [2], suggesting that BET inhibitors may be effective against NMCs with clinical trials actively evaluating BET inhibitors in NMC patients (Table 2). Significantly, a recent report evaluated anti-tumor activity in four advanced NMC patients treated with the oral BET inhibitor OTX015/MK-8628 on a compassionate basis, and demonstrated rapid tumor regression and symptomatic relief in two patients [22]. Significantly, the OS of these two patients was 18 and 19 months, much longer than the median OS of 6.7 months previously reported for advanced NMC patients [20].

**Table 2:** Clinical Trials of BET inhibitors in Solid Tumors

Drug	Cancer	Phase	Trial (accessed clinicaltrials.gov on 02/10/2106)
BAY1238097	Advanced solid tumors	1 (ongoing, but not recruiting)	NCT02369029
BMS-986158 +/- Paclitaxel	OvC, SCLC, TNBC	1/2 (recruiting)	NCT02419417
GSK525762	NMC, SCLC, NSCLC, CRC, NB, CRPC, TNBC, ER+ BC	1 (recruiting)	NCT01587703
GSK2820151	Advanced solid tumors	1 (not yet open)	NCT02630251
INCB054329	Advanced solid tumors	1/2 (recruiting)	NCT02431260
OTX015	GBM	1/2 (terminated)	NCT02296476
OTX105/ MK-8628	NMC, TNBC, CRPC, PDAC NSCLC	1 (ongoing, but not recruiting)	NCT02259114
TEN-010	Advanced solid tumors	1 (recruiting)	NCT01987362

BC, breast cancer; CRC, colorectal cancer; CRPC, castrate resistant prostate cancer;

GBM, glioblastoma; NB, neuroblastoma; NMC, nut midline cancer; NSCLC, non-small

cell lung cancer; OvC, ovarian cancer; PDAC, pancreatic ductal adenocarcinoma; SCLC,

small cell lung cancer; TNBC, triple negative breast cancer.

### BET inhibitors and breast cancer

#### Treatment of tamoxifen-resistant breast cancer

Breast cancer is currently the second leading cause of cancer death in women. The 5-year survival for breast cancer patients is > 90%, but as the most diagnosed cancer in women, a significant number of patients will ultimately die of their disease [23]. The estrogen-receptor (ER)-positive breast cancers represent ~70% of all breast cancers, and the selective ER modulator tamoxifen remains a mainstay of treatment for these patients [24]. While tamoxifen is effective in reducing recurrence and death from breast cancer [25-27], most tumors eventually develop tamoxifen resistance even while maintaining their reliance on estrogen-mediated signaling [28, 29]. Significantly, BET proteins contribute to tamoxifen resistance by recruiting WHSC1, a histone H3K6 methyltransferase, to the *ERα* gene with inappropriate modulation of expression [11]. BET proteins directly interact with WHSC1, and knockdown of BET proteins decreases ERα expression and downstream signaling [11]. Importantly, tamoxifen-resistant cell lines are more sensitive than parental cell lines to the BET inhibitor JQ1 [11]. JQ1 causes persistent suppression of both ERα and c-MYC in tamoxifen-resistant cells, while similar treatment in parental cell lines results in re-expression of both ERα and c-MYC [11]. JQ1 moderately inhibits tumor growth in xenograft mice harboring tamoxifen-resistant cells, but JQ1 in combination with fulvestrant, a selective ER degrader, has synergistic antitumor activity with potent inhibition of tumor cell proliferation in the same model system [11]. Furthermore, ERα protein levels are significantly down regulated in tumors treated with both fulvestrant and JQ1 [11].

#### Treatment of everolimus-resistant breast cancer

The mTOR pathway has also been shown to mediate resistance to anti-estrogens in women with ER-positive breast cancer [30]. Everolimus, an allosteric inhibitor of mTOR complex 1, has been approved in combination with exemestane for treatment of ER+/Her2- breast cancer patients who have progressed on treatment with anastrozole or letrozole [31]. This combination increased progression-free survival (PFS) compared to exemestane alone [31]. However, despite initial efficacy, breast cancer cells can develop acquired resistance to everolimus. In one long-term estrogen deprivation model, resistance occurred through increased c-MYC expression mediated by BRD4 [32]. Notably, down-regulation of c-MYC using siRNA or the BET inhibitor JQ1 restored everolimus sensitivity, while a combination of everolimus and JQ1 led to synergistic growth inhibition in 3D Matrigel cultures and xenograft models [32].

#### Treatment of lapatinib-resistant breast cancer

The HER2 oncogene is amplified or overexpressed in ~25% of breast cancers and serves as the primary driver of tumor cell growth in the majority of HER2+ tumors [33]. There are several FDA approved agents for the treatment of HER2+ breast cancers, including monoclonal antibodies and the small molecule inhibitor lapatinib [34]. Unfortunately, acquired resistance to HER2-directed therapies is a clinical challenge for patients with advanced HER2+ disease [35]. Resistance to lapatinib can result from upregulation of HER3 and from activation of multiple tyrosine kinases [35], suggesting that tumor cells can reprogram their signaling kinome to overcome the inhibitory effects of lapatinib. Significantly, BET inhibitors can suppress the kinome reprogramming response seen in lapatinib-treated breast cancer cells [36]. JQ1 caused greater suppression in genes upregulated by lapatinib than in genes unaffected by or even down regulated by lapatinib, suggesting that JQ1 preferentially modulates lapatinib-responsive gene expression [36]. Furthermore, clonogenic growth assays demonstrated that dual treatment with lapatinib and JQ1—but not monotherapy with JQ1 alone—blocked the growth of lapatinib-resistant cells [36].

#### Treatment of triple-negative breast cancer

The triple negative breast cancers (ER-, PR-, and HER2-; TNBCs) account for ~20% of breast cancers [37, 38]. These tumors are often among the most aggressive breast cancers and are treated primarily with chemotherapy. In a recent screen of breast cancer cell lines, TNBC lines were found to be particularly sensitive to BET inhibitors compared to luminal and HER2+ breast cancer lines [39]. The BET inhibitor JQ1 or BRD4 siRNA blocked growth of TNBC cell lines by decreasing proliferation and inducing apoptosis and/or senescence [39], while similar treatments inhibited tumor growth in TNBC mouse xenografts [39]. Mechanistically, JQ1 treatment preferentially repressed genes associated with super-enhancers [5, 40]. In this setting, JQ1 did not consistently repress c-MYC, but treatment with JQ1 resulted in deregulation of transcriptional pathways important for cell survival, proliferation and invasion [39].

Overall, emerging evidence suggests that in patients with breast cancer, BET inhibitors may be of distinct therapeutic benefit in a range of disease subtypes through modulating acquired resistance to estrogen blockade in ER+ disease; enhancing the known therapeutic benefits of mTOR inhibitors; allowing for more durable response in combination with lapatinib in patients with HER+ disease; and decreasing growth of TNBCs.

### BET inhibitors and prostate cancer

Prostate cancer is the most commonly diagnosed cancer in men in the US. Significant progress has been made in the treatment options for prostate cancer patients, but over 27,000 men will die of the disease in 2015 in the US alone [23]. The mainstay of treatment of advanced prostate cancer involves targeting androgen receptor (AR) signaling through one of several different drugs that either block androgen production (e.g., abiraterone) or block the AR itself (e.g., enzalutamide) [41]. Enzalutamide is currently approved by the FDA for the treatment of castrate resistant prostate cancer (CRPC) both following and prior to docetaxel chemotherapy [42, 43]. Unfortunately, durable responses to enzalutamide are limited, so there is increasing interest in identifying additional targets for the treatment of CRPC.

BET inhibitors are effective in CRPC through targeting of the AR signaling network [10]. JQ1 blocks proliferation, induces apoptosis, and represses expression of anti-apoptotic factors in AR+ cells while also reducing transcription of AR target genes [10], indicating that BET proteins are involved in AR-mediated transcriptional programs. Significantly, JQ1 reduces recruitment of the AR to AR-responsive genes to nearly the same extent as the direct AR antagonist enzalutamide [10]. Moreover, in mouse studies, JQ1 does not affect normal prostate growth or testosterone levels even while decreasing growth of CRPC tumors [10]. JQ1 is more effective than enzalutamide in blocking tumor growth, and in contrast to enzalutamide-treated mice, animals treated with JQ1 do not develop liver or bone metastasis [10].

Recently, it was also shown that BET inhibitors are effective against CRPC cell lines that have become resistant to enzalutamide [44]. JQ1 decreases protein levels of AR-variant 7, previously identified as one of the major drivers of resistance to androgen-deprivation therapy (ADT) [45]. Significantly, BET inhibitors display enhanced efficacy when combined with enzalutamide *in vivo* [44]. Together, these studies demonstrate that combining BET inhibitors with anti-androgens could result in more durable therapeutic responses in patients with CRPC by subverting resistance mechanisms to ADT.

### BET inhibitors and lung cancer

#### Treatment of non-small cell lung cancer

Lung cancer is the most frequent cause of cancer mortality worldwide [46], with non-small cell lung cancer (NSCLC) accounting for approximately 85 percent of lung cancers in the US [23]. Advanced NSCLC is now treated based on genotype, with first-line therapy for a growing number of patients now an oral tyrosine kinase inhibitor instead of chemotherapy. However, long-term durable disease control is not yet reality for the majority of advanced NSCLC patients, regardless of genotype, because of the challenge of acquired resistance [47]. Preclinical studies in a range of lung adenocarcinoma cell lines harboring either *KRAS* or *EGFR* mutations suggest that BET inhibitors may have clinical efficacy in the treatment of NSCLC [15]. In these cell lines, JQ1 treatment led to decreased proliferation, cell cycle arrest, and induction of apoptosis mediated by the repression of FOSL1, a component of the FOS-JUN transcription factor complex [15].

Perhaps even more significant, JQ1 has also been shown to specifically have activity in preclinical models of *KRAS* mutant NSCLC. Although *KRAS* mutations are found in an estimated 30% of lung adenocarcinomas, there is not yet an effective targeted therapy for the majority of these patients [48]. A murine co-clinical trial demonstrated that concurrent mutations in *LKB1* or *TP53* may help mediate differential response to concurrent chemotherapy and MEK inhibition in these tumors, [49] and interestingly, co-expression of mutant LKB1 also limits the effectiveness of JQ1 in *KRAS* models [50]. *LKB1* encodes a serine-threonine kinase that directly phosphorylates and activates AMPK, a central metabolic sensor [51]. JQ1 and BRD4 knockdown induces apoptosis in *KRAS* mutant cell lines but not in the presence of concurrent *LKB1* mutation [50]. Similarly, in a transgenic mouse model, JQ1 decreased proliferation of *KRAS* mutant tumors but not of mutant *KRAS/LKB1* tumors [50], further demonstrating that *LKB1* may be a key modulator of the efficacy of BET inhibitors in *KRAS* mutant NSCLC.

#### Treatment of small cell lung cancer

Small cell lung cancer (SCLC) accounts for ~13-15% of lung cancer cases in the US [52]. SCLC has a high recurrence rate even after definitive chemotherapy, and the 5 year survival rate for SCLC patients is < 5% [52]. In a recent screen of 83 lung tumor cell lines in a cell proliferation assay, SCLC lines were found to be exquisitely sensitive to BET inhibitors even though c-MYC levels were unaffected by JQ1 in the sensitive SCLC lines [53]. Instead, JQ1 blocked BRD4 binding to the enhancer of achaete-scute homolog-1 (ASCL1), thereby decreasing ASCL1 expression levels. ASCL1 is a transcription factor important for development of neuroendocrine progenitor cells [53]. In addition, siRNA targeting ASCL1 also decreased proliferation and phenocopied the effects of JQ1 in the sensitive cell lines. Significantly, over 50% of human SCLC tumor specimens were found to overexpress ASCL1 [53], suggesting that human SCLC tumors with increased ASCL1 expression may benefit from treatment with BET inhibitors.

### BET inhibitors and gastrointestinal cancers

#### Treatment of pancreatic cancer

Pancreatic ductal adenocarcinoma (PDAC) is currently the 4^th^ leading cause of cancer-related death in the US and is projected to become the 2^nd^ leading cause of cancer-related death by 2020 [23, 54]. Current standard-of-care for advanced PDAC is cytotoxic chemotherapy, but the success of current drug therapies is severely limited [55, 56]. We have shown that BET inhibitors are effective against chemotherapy-resistant PDAC cells, in part through repression of HMGA2 [16], a non-histone DNA-binding nuclear protein involved in chromatin remodeling and gene transcription [57, 58]. JQ1 decreased HMGA2 in cell lines isolated from mouse models of pancreatic cancer [59], while also decreasing growth of mouse cell lines *in vitro* with decreased proliferation and increased apoptosis in mouse tumors *in vivo* [59]. Moreover, JQ1 suppressed growth of PDAC tumors in patient-derived xenograft (PDX) mouse models [60]. Treated PDX tumors did not show consistent changes in c-MYC levels, but expression profiling identified CDC25B—a regulator of cell cycle progression—to be the major target of JQ1 in this setting [60]. Finally, BET inhibitors were found to suppress PDAC growth and improve survival in the transgenic KPC (Kras/p53) PDAC mouse model [61]. In this model, JQ1 treatment repressed Myc and attenuated inflammation *in vivo*. JQ1 and siRNA targeting BRD4 both decreased IL-6 production and inhibited Stat signaling [61], pathways previously found to mediate PDAC progression in mouse models [62, 63]. Overall, these reports strongly indicate that BET inhibitors may be effective against PDAC.

#### Treatment of colon cancer

Colon cancer is currently the 2^nd^ leading cause of cancer-related death in the US, and patients with advanced colon cancer have a median overall survival of approximately 2-3 years based primarily upon chemotherapy-based treatment regimens [23, 64]. Recently, an array-based CRISPR screen identified BRD4 as a driver of proliferation and mediator of de-differentiation in colon cancer [65]. BRD4 knockdown decreased proliferation *in vitro* and decreased tumor growth in xenograft mouse studies [65]. BRD4 knockdown also repressed c-MYC in xenograft studies and induced differentiation into ‘normal-like’ intestinal epithelium [65]. Significantly, a subset of colon cancer cell lines with a CpG island methylator phenotype (CIMP) were particularly sensitive to JQ1 treatment and to JQ1-induced c-MYC repression [65]. Approximately 20% of human colon cancer tumors arise through the CIMP pathway, and these tumors often have poor outcomes [66]. BET inhibitor treatment of CIMP(+) cell lines repressed expression of colon cancer-associated transcript 1 (CCAT1), a long non-coding RNA known to be transcribed off the *c-MYC* superenhancer in colon cancer [65]. Interestingly, CCAT1 expression also predicted for JQ1 sensitivity not only in colon cancer cell lines, but also in lung and pancreatic cancer cell lines [65].

#### Treatment of hepatocellular cancer

Worldwide, hepatocellular cancer (HCC) is the second leading cause of cancer-related death in men [46]. Although the multi-targeted small molecule tyrosine kinase inhibitor sorafenib is approved for the treatment of advanced HCC [67], OS remains less than a year [23]. Significantly, BRD4 is overexpressed in human HCC tumors, and treatment with JQ1 decreases proliferation of HCC cell lines and primary cells isolated from human HCC tumors [68]. JQ1 also blocks growth of HCC tumors in xenograft mouse models [68]. In HCC cells, JQ1 induces cell cycle arrest primarily through decreasing c-MYC expression and increasing expression of p27 [68], along with induction of apoptosis through upregulation of the pro-apoptotic gene BIM [68]. Overall, these findings suggest that BET proteins may be potential therapeutic targets in the treatment of HCC.

### BET inhibitors and brain tumors

#### Treatment of glioblastoma

Glioblastoma (GBM) is the most common primary brain cancer in adults with a median OS of 15-17 months and a 5-year survival of less than 5% [69, 70]. GBM has been classified into different subgroups based upon complex genetic and signaling aberrations [71, 72], and BET inhibitors have been shown to have efficacy in a range of GBM models reflecting these different subgroups [73, 74]. JQ1 decreased proliferation of both CD133+ GBM stem cells and non-stem cancer cells while promoting apoptosis, decreasing c-MYC and BCL-XL levels, and increasing p21 levels [73]. JQ1 also blocked GBM progression in an orthotopic tumor model [73].

BET inhibitors have also been evaluated in GBM tumors with aberrant EGFR signaling [74]. *EGFR* is mutated or amplified in > 50% of GBM tumors [71], with the EGFRvIII mutation resulting in ligand-independent activation of EGFR signaling [75]. Significantly, EGFRvIII sensitizes GBM cells to JQ1, with JQ1 inducing apoptosis and suppressing EGFRvIII-dependent tumor growth *in vitro* and in xenograft orthotopic mouse model [74]. Mechanistically, in GBM cells EGFRvIII induces SOX9 and FOXG1, which in turn collaborate to activate an oncogenic gene regulatory program [74]. SOX9 and FOXG1 also regulate expression of BRD4 with subsequent regulation of c-MYC expression to promote tumor growth [74]. Together, these results suggest that BET inhibitors may have efficacy in GBM, particularly GBM patients whose tumors harbor an EGFRvIII mutation.

#### Treatment of medulloblastoma

Medulloblastoma is the most common malignant brain tumor of childhood [76]. Transcriptional profiling studies have identified four distinct molecular subgroups of medulloblastoma: Wnt, Sonic hedgehog (Shh), Group 3, and Group 4 [77]. Group 3 medulloblastoma is often associated with amplification of *c-MYC* and has the worst overall prognosis, with 5-year OS rates of only 50% [76, 77]. Notably, several studies have shown that JQ1 has efficacy in *c-MYC*-amplified medulloblastoma [78-80]. Treatment with JQ1 decreased c-MYC expression and inhibited c-MYC-associated transcriptional targets [78-80]. JQ1 also suppressed stem cell-associated signaling in medulloblastoma cells and inhibited medulloblastoma tumor cell self-renewal [80]. Furthermore, JQ1 treatment reduced tumor growth and prolonged survival in mice harboring medulloblastoma xenografts [78-80].

BET inhibitors have also been found to be effective against the Shh subgroup of medulloblastoma [76]. In canonical Hedgehog (Hh) signaling, Hh ligands bind to the cell-surface receptor Patched, triggering a Smoothened (SMO)-dependent signaling cascade that results in activation of GLI transcription factors and transactivation of Hh target genes [81]. While SMO inhibitors have shown efficacy against medulloblastoma [82, 83], tumors eventually develop resistance to SMO inhibitors [84, 85]. Recently, studies identified that BRD4 directly occupies GLI1 and GLI2 promoters, and the BET inhibitors JQ1 and I-BET151 decreased expression of GLI1, GLI2 and GLI-target genes in medulloblastom [86, 87]. JQ1 inhibited cell viability and proliferation in SMO-inhibitor resistant Hh-driven medulloblastoma cell lines [86], while BET inhibitors also decreased Hh-driven medulloblastoma in xenograft mouse models [86, 87]. Together, these results suggest that BET inhibitors may be effective in both Shh and Group 3 medulloblastomas.

## POTENTIAL TOXICITIES OF BET INHIBITORS

Silencing of BRD4 in transgenic mouse models suggests that treatment with potent BET inhibitors will likely have clinical toxicities [88]. Sustained BRD4 knockdown was found to induce epithelial hyperplasia and follicular skin defects that were rapidly reversed when BRD4 was restored in the mouse model [88]. BRD4 knockdown also caused loss of multiple cell types in the intestine, including a reduction in the number of functional stem cells [88]. Similarly, treatment of wild-type mice with a small molecule BET inhibitor suppressed intestinal stem cell differentiation [89]. However, the intestinal changes were reversible in both the BRD4 knockdown experiments and the BET inhibitor mouse studies, suggesting that these potential toxicities could be managed with appropriate dose scheduling on a human clinical trial.

Mouse studies have also suggested that BET inhibitors may exacerbate toxicities seen with concurrent radiation and chemotherapy treatment [88, 89]. Transgenic mice with BRD4 knockdown were more likely to develop radiation damage to the intestines, with delay in repair and recovery of normal bowel function [88]. In addition, mice treated with a BET inhibitor demonstrated increased apoptosis in the intestine when co-treated with gemcitabine [89]. BET inhibition has also been shown to exacerbate colitis in mice treated with dextran sodium sulfate [90]. There is clearly potential for synergistic toxicities when BET inhibitors are combined with other therapies, and this will have to be carefully considered during clinical trial design. However, these synergistic effects were also reversible [88, 89], further emphasizing the importance of clinical trial design for BET inhibitors used in combination studies.

## MECHANISMS OF RESISTANCE TO BET INHIBITORS

As the effectiveness of targeted therapies can be limited by *de novo* resistance or by subsequent development of resistance [91], there has been increasing interest in characterizing mechanisms of resistance to BET inhibitors. This is particularly important as a better understanding of the mechanisms of resistance may identify which patients and types of cancers should be treated with BET inhibitors, and may allow for identification of additional therapeutic targets that may extend the efficacy of BET inhibitors. However, until recently little was known about the mechanisms by which cancer cells developed resistance to BET inhibitors.

### Re-expression of MYC

We have shown that pancreatic cancer cells developing resistance to JQ1 were also resistant to other BET inhibitors and to BRD4 down regulation [92]. Our work demonstrated that the JQ1-resistant cells upregulated c-MYC through increased binding of GLI2 to the *c-MYC* promoter, allowing continued cell growth in 3D collagen. Significantly, targeting GLI2 re-sensitized pancreatic cancer cells to BET inhibitors and BRD4 down regulation [92]. Consistent with our findings, leukemia cells have also been shown to upregulate c-MYC levels during the development of resistance to BET inhibitors [93, 94]. Resistant cells also appeared to contribute to expansion of the leukemia stem cell population [93]. Transcriptional profiling of the resistant cells demonstrated activation of the WNT transcriptional program, thus facilitating c-MYC re-expression [93, 94]. Notably, WNT-β-catenin signaling has previously been shown to be important for cancer stem cell maintenance [95], and blocking WNT targets in this model not only re-sensitized the leukemia cells to JQ1 but also led to re-suppression of c-MYC [93, 94]. Activation of the WNT pathway in leukemia cells *in vivo* was also found to drive *de novo* resistance to BET inhibition [93]. Together, these results demonstrate that in some models, resistant cells continue to rely on c-MYC to drive proliferation, but in the face of BET inhibition, resistant cells will shift from BRD4-mediated expression of MYC expression to alternative pathways, including GLI2 or WNT-β-catenin signaling, in order to maintain MYC levels.

### Bromodomain-independent role of BRD4

In contrast to the resistance mechanism identified in pancreatic cancer and leukemia cells [92-94], TNBC cells developing resistance to BET inhibitors continue to rely on BRD4 for ongoing proliferation [39]. Resistant cells remain sensitive to BRD4 knockdown, suggesting that resistant cells activate a bromodomain-independent role of BRD4 with subsequent recruitment of BRD4 to enhancers [39]. Resistant cells also demonstrate increased binding of BRD4 to MED1 in a bromodomain-independent manner that is unaffected by BET inhibitors [39]. Finally, resistant cells demonstrate hyperphosphorylation of BRD4 as a result of decreased activity of the phosphatase PP2A and resulting in increased binding of BRD4 to MED1 [39].

### Activation of alternative signaling pathways

Using a whole-genome shRNA screen of 77 breast cancer cell lines to identify cancer drivers, BRD4 was identified as a potential target in luminal breast cancer [96]. Luminal/HER2+ cells were more sensitive to BRD4 knockdown than basal breast cancers [96]. Clinically, luminal breast cancer cells are typically ER+/PR+, [97] while basal breast cancer cells are usually triple-negative [37, 98]. Surprisingly, many of the luminal/HER2+ breast cancer cell lines that were sensitive to BRD4 knockdown were subsequently found to be resistant to JQ1 treatment, suggesting that BRD4 also has a bromodomain-independent role in this cell type [96]. Intriguingly, a strong correlation was seen between JQ1 resistance and concurrent PIK3CA mutation. Overexpression of PI3KCA in sensitive breast cancer cells conferred resistance to JQ1, while treatment with a PI3KCA inhibitor sensitized resistant cells to JQ1 [96]. Using mTOR inhibitors to block downstream PI3K signaling sensitized resistant cells to JQ1 *in vitro* and *in vivo* [96]. Conversely, combining BET inhibitors with PI3K inhibitors can sustain PI3K inhibition and enhance cell-killing [99]. Significantly, BET inhibitors can also enhance the therapeutic benefit of mTOR inhibitors in breast cancer cells [32]. Overall, these results suggest that targeting PI3K/mTOR signaling may help sensitize JQ1-resistant cells to BET inhibitors.

## CONCLUSIONS

A growing body of research has now demonstrated that BET inhibitors have a significant anti-tumor effect in a range of solid tumors and represent an exciting new avenue of targeting tumor growth through modulation of transcriptional programming. Some tumors, including triple negative breast cancer and small cell lung cancer [39, 53], are particularly sensitive to BET inhibitors. Patients with these tumors may be ideal candidates for BET inhibitor trials, and several ongoing studies are actively enrolling patients with these particular cancers (Table 2). In addition, BET inhibitors may also have a role in preventing or overcoming acquired resistance to targeted therapies in patients whose treatment options currently include FDA-approved therapies [10, 32, 36, 44, 99]. Moving forward, it will be important to determine whether BET inhibitors can extend response to lapatinib in breast cancer patients or to enzalutamide in prostate cancer patients. For many tumors, effective use of BET inhibitors will likely require a combination approach with other targeted and epigenetic therapies, and this in turn will require careful analysis of trial design and dosing schedules to minimize overlapping toxicities. Finally, as we further elucidate the resistance mechanisms that govern the overall response to BET inhibitors [39, 92-94], targeting these resistance pathways will provide new opportunities to further increase the clinical efficacy of BET inhibitors.
